# Application of Virtual Reality Technology in Clinical Practice, Teaching, and Research in Complementary and Alternative Medicine

**DOI:** 10.1155/2022/1373170

**Published:** 2022-08-11

**Authors:** Huifang Guan, Yan Xu, Dexi Zhao

**Affiliations:** ^1^College of Traditional Chinese Medicine, Changchun University of Chinese Medicine, Changchun 130117, China; ^2^College of Pediatrics, Henan University of Chinese Medicine, Zhengzhou 450000, Henan, China; ^3^Department of Encephalopathy, The Affiliated Hospital of Changchun University of Chinese Medicine, No. 1478 Gong-Nong Road, Changchun, Jilin 130021, China

## Abstract

**Background:**

The application of virtual reality (VR) in clinical settings is growing rapidly, with encouraging results. As VR has been introduced into complementary and alternative medicine (CAM), a systematic review must be undertaken to understand its current status.

**Aim:**

This review aims to evaluate and summarize the current applications of VR in CAM, as well as to explore potential directions for future research and development.

**Methods:**

After a brief description of VR technology, we discuss the past 20 years of clinical VR applications in the medical field. Then, we discuss the theoretical basis of the combination of VR technology and CAM, the research thus far, and practical factors regarding usability, etc., from the following three main aspects: clinical application, teaching, and scientific research. Finally, we summarize and propose hypotheses on the application of VR in CAM and its limitations.

**Results:**

Our review of the theoretical underpinnings and research findings to date leads to the prediction that VR and CAM will have a significant impact on future research and practice.

**Conclusion:**

Although there is still much research needed to advance the science in this area, we strongly believe that VR applications will become indispensable tools in the toolbox of CAM researchers and practitioners and will only grow in relevance and popularity in the era of digital health.

## 1. Introduction

The rapid evolution of digital technology has allowed for novel and creative solutions across medical disciplines in recent years. Among these technologies, virtual reality (VR) has become a potentially powerful adjunct. VR affords the opportunity to create highly realistic, interactive, and systematically controlled stimulus environments that users can be immersed in and interact with for human testing, training, teaching, and treatment environments that allow for the precise control of complex, multisensory, and dynamic 3D stimulus presentations [1].

In recent years, complementary and alternative medicine (CAM) has become more popular worldwide, and the number and proportion of its uses continue to grow [2]. The combination of VR and CAM has received extensive attention. Several recent studies, reviews, and meta-analyses have shown that VR plays a positive role in CAM treatments such as meditation, hypnosis, palliative therapy, tai chi (TC), qigong, acupoint sticking therapy, aromatherapy, and yoga [3–10]. In addition, VR has helped clinicians overcome barriers in education [11–24] and research [25, 26] during the coronavirus disease 2019 (COVID-19) pandemic. To some extent, VR opens the door to a new generation of application programs in CAM.

The COVID-19 pandemic has become one of the largest global health crises of our time [27]. Excessive pressure on health care systems has prompted medical resources around the world to be redirected to stop the spread of COVID-19 and treat severe cases. In fact, while there have been hundreds of millions of cases of COVID-19 worldwide, the pandemic has brought about social problems and thus has forced the integration and development of VR technology in the field of CAM.

First, many patients have not been able to receive timely help due to the impact of COVID-19. Therefore, facilities offering services such as CAM have had to adapt their service offerings and develop virtual medicine strategies to ensure that their patients continue to receive necessary treatment.

Second, there is a high level of transmission of SARS-CoV-2, the virus that causes COVID-19; as a result, countries worldwide have imposed rigorous public health measures, such as quarantines. This has involved the suspension of medical school classes globally, resulting in students not being able to rotate at their institutions [28]. This results in medical students having less clinical experience, while varied and rich clinical experiences are the cornerstone of medical students' growth. This requires an unprecedented change in the way the medical education sector provides clinical instructions, in line with efforts aimed at prioritizing the safety and slowing the spread of the virus. Several studies have attempted to fill this gap by applying VR to medical education and training to support physician learning during social distancing [11, 13, 15, 18, 22, 23].

Third, COVID-19 has led to high levels of burnout and mental illness in medical students [29]. Mind-body interventions such as VR-based yoga [9] and mindfulness meditation [30] can be used as successful tools for stress management and the reduction of burnout rates and anxiety in resident physicians. VR can offer an immersive environment to enhance the user's experience and prevent distractions [31]. Research studies showed that 10 minutes of VR therapy was similar in effect to reducing work by 1.6 hours per week with regard to reductions in emotional exhaustion [30]. To this end, an important benefit of VR is the minimal time commitment necessary, allowing medical residents to benefit from decreased burnout without losing important educational opportunities [30].

Fourth, the application of VR has complemented strict preventive measures to reduce the infection rate of medical workers on the front lines of the COVID-19 pandemic.

Finally, during the COVID-19 pandemic, the burden on the medical system and medical costs have increased, which has become an emerging problem in the medical system. The application of VR in CAM can reduce the need for face-to-face consultation, thereby reducing the use and transportation of medical resources (such as protective clothing).

Even as countries and systems adapt to the new normal after the COVID-19 pandemic, many virtual systems built to meet short-term needs will eventually evolve into long-term trends and solutions. Therefore, a systematic review of the application of VR in the field of CAM can provide inspiration and reference for research on and development of related projects in the future.

Some systematic reviews have been published, but their scope only partially overlaps with that of this paper. For example, some systematic reviews examined only VR and meditation or VR and hypnosis, without a comprehensive review of VR and the entire field of CAM; other reviews were published 5 years ago and therefore lack recent references. This paper expands on previous findings by providing a broader and updated overview of the potential of VR in CAM.

This review briefly presents evidence on how VR can be rationally used in conjunction with CAM in a range of settings, including clinical, educational, and scientific research settings. This article presents the potential advantages and disadvantages of using VR in CAM, as well as practical recommendations on how to incorporate VR into CAM.

## 2. What Is VR?

Before one can explore VR, it is useful to consider how it is defined. The term “virtual reality” itself is credited to Jaron Lanier, who, in 1989, developed a full-body suit of sensors for body movement recordings, a technique that is extensively used in film and game productions [32].

However, the technology was not sufficiently mature in the 1990s. As underlying VR-enabling technologies and methods (e.g., computational speed, computer graphics, panoramic video, audio/visual/haptic displays, natural user interfaces, tracking sensors, speech and language processing, artificial intelligence, virtual human agents, and authoring software) have continued to evolve [1], the definition of VR has also evolved alongside advancements in technical capabilities, from an early stage of large projection rooms to current consumer products that use high-resolution head-mounted displays (HMDs) [33]. Users of VR technology wear an HMD with a close-proximity screen that creates a sensation of being transported into lifelike, three-dimensional worlds [34], and the use of HMDs has three key characteristics: presence, immersion, and interactivity [35]. Presence mainly refers to the user's sense of immersion. The sense of immersion refers to the use of multiple senses, such as hearing, vision, touch, taste, and smell. Finally, interactivity is another key component of VR. Human-computer interaction allows people to operate VR systems at will and obtain the most realistic feedback from the environment during the operation. Multimodal stimulus control is important for inducing a sense of ‘presence' in virtual environments, which is believed to be of crucial importance for the effectiveness of VR training [36]. The most commonly used forms of sensory stimulation are visual and auditory displays [36]. Additionally, VR systems may provide limited but compelling haptic feedback to simulate the sensation of forces, surfaces, and textures when users interact with virtual objects [36].

## 3. How Does VR Technology Work in a Medical Setting?

It is the abovementioned characteristics of VR technology that make it loved by many people and widely used in many fields, such as the medical field. To date, VR has successfully been applied in many clinical settings [1], such as helping to treat anxiety disorders [37, 38], alleviating fear [39], managing pain [33, 34, 40], supporting physical recovery [41], and preventing falls in elderly individuals [42]. Furthermore, an interactive training system for public health emergency preparedness for major emerging infectious diseases based on VR should be established [43].

Likewise, VR has revolutionized medical education [44]. Opportunities for repeated exposure and hands-on experience are important for medical students. However, this puts patients at an increased risk. Therefore, VR is emerging as a necessary augmentation to conventional learning [45–47]. For example, VR can help train students in anatomy [48, 49], helping physicians optimize preoperative and intraoperative decision-making [50, 51]. For example, after VR simulation training in endoscopy, trainees were found to improve in areas such as the comprehensive assessment of technical and nontechnical skills and patient comfort [52].

In scientific research, the use of VR to create an integrative web-based VR system to explore the macromolecular structure is a new trend [53], and VR can be further used for novel drug development, such as drug discovery and rational drug design [54].

## 4. What Is CAM?

The term “complementary and alternative medicine” refers to interventions that are not part of conventional medical care but are provided alongside it as a supplement [55]. There is a broad range of interventions that fall under the realm of CAM, including ancient medicine traditions such as ayurvedic or traditional Chinese medicine, acupuncture, meditation, hypnotherapy, yoga, TC, and music intervention [55, 56]. Today, CAM has widespread use worldwide and is applied to various diseases and conditions, especially intractable diseases and conditions such as cancer, pain [57], and chronic diseases [58].

## 5. Clinical Application

### 5.1. Meditation

Meditation is a mental practice aiming to improve the psychological capacity of self-regulation regarding attention, awareness, and emotion [59]. Studies have found evidence of the positive effects of meditation on health and well-being, but the difficulty of learning and engaging in meditation practice has been identified as a major barrier [60]. VR technology may facilitate meditation practice by immersing users in a distraction-free and calming virtual environment [60]. Today, VR and meditation therapy have been applied to a range of disorders and conditions, including pain [60–62], depression [63], anxiety disorders [3, 63, 64], sleep disorders [65], posttraumatic stress disorder [66], and pressure [60].

Regarding pain management, clinical studies have validated the effectiveness of VR as a facilitator of meditation practice in patients with acute pain [62], chronic pain [60], and opioid tolerance or opioid use disorder [61, 62]. Further neurobiological research studies found that scores for pain, opioid craving, anxiety, and depression decreased after each intervention session (relative to before the session) [61]. In addition, salivary cortisol (but not CRP) levels were found to decrease from pre- to postsession [61]. Based on pre- to postintervention fMRI assessments, painful task-related left postcentral gyrus (PCG) activation was found to decrease [61]. At baseline, the PCG showed positive connectivity with other regions of the pain neuromatrix, but this pattern changed postintervention [61]. The results of this feasibility study suggest that a VR-based meditation intervention is a promising approach for reducing pain scores and modulating pain neuromatrix activity and connectivity among patients with opioid use disorder [61].

The prolonged illness and recovery time of COVID-19, coupled with infection prevention measures that make on-site family visits or movement between hospital units difficult or contraindicated, present a range of challenges for patients hospitalized with COVID-19, such as social isolation, disability, neurologic sequelae, adjustment-related anxiety, depression, stress, sleep disorders, and posttraumatic stress disorder [67]. It has been suggested that novel VR-based meditation interventions could be used as a comprehensive recovery program for COVID-19 [3, 63–67] and as successful stress management tools to reduce burnout rates among residents [30].

### 5.2. Hypnosis

Hypnosis is defined as “a state of consciousness involving focused attention and reduced peripheral awareness characterized by an enhanced capacity for response to suggestion”. Hypnosis has been shown to be efficacious for a range of clinical conditions, such as relief of pain [68, 69]. However, there is a universal agreement that individual differences in hypnotizability exist, meaning that not all individuals are able to enter a hypnotic state, thereby limiting the clinical utility of this technique [70]. In fact, those lacking imaginative absorption-like traits have often shown little or no benefits in response to hypnosis in studies [10]. However, if the visual and auditory stimuli provided by VR can be experienced by individuals with low hypnotic susceptibility, these individuals have to rely less on their own imagination, which improves the intervention effect [10].

With attention mechanisms as a common denominator, the potential for synergy between these two modalities in VR and hypnosis is significant for several reasons. First, hypnotic suggestions may help an inhibited patient relax and immerse himself or herself in a virtual world. Furthermore, hypnotic suggestions can be used to deepen a patient's sense of presence in the virtual world [71].

Currently, a new technique called VR hypnosis (VRH), which encompasses a combination of both tools combined with VR hardware/software and hypnosis induction [72], is regularly used to treat anxiety and pain [73]. This method immerses the patient in a relaxed, peaceful environment. It represents a noninvasive way to reduce preoperative stress levels without side effects and without the need for additional medical or support staff. In parallel experiments, the combined effect of hypnotic analgesia and VR pain distraction was stronger than that of VR distraction alone [74]. The combination of hypnosis and VR can be used to treat a variety of types of pain, such as pain following traumatic injuries [75] or spinal cord injury-associated neuropathic pain [76]; this combination has been widely used to relieve preoperative anxiety in preoperative patients, such as beforehand surgery under axillary plexus block [77] or cardiac surgery [78]. In a review that included 8 studies on VRH, short-term results showed significant reductions in pain intensity, unpleasant pain, time spent thinking about pain, anxiety, and opioid craving levels, and improved short-term quality of life in patients [72]. In contrast, the Violeta Enea study found that although hypnosis + VR had the same efficacy as hypnosis alone and VR alone, it appeared that their combination did not have an additive effect and that the two interventions might even interfere with each other [79].

### 5.3. Palliative Care

During COVID-19, strict inpatient visitation restrictions to prevent infection have meant that many people have died alone in hospitals [80]. With limited resources and a rapidly increasing number of patients, the desperate race to fight to preserve life has understandably but regrettably led to inattention to those dying [81]. Existential pain and psychological barriers for patients and their families may last a lifetime [81]. To help meet this challenge, several institutions have used VR as a supplement to palliative care during the COVID-19 pandemic [81]. Using VR to have conversations with relatives of patients in palliative care at the end of life makes the patient and family feel like they are in the same room, promotes connection between patients and their families, and creates opportunities for final contact before death [5, 82, 83]. Virtual palliative care can also help address challenges and barriers to providing such care, including geographic barriers, clinician staffing, and outreach to underserved populations [84]. Some health systems have introduced virtual palliative care to meet growing demands [85, 86] and to expand their insurance coverage during the COVID-19 pandemic [87].

During the COVID-19 crisis, a New York City hospital virtually trained hospitalists practicing remotely to partner with on-site clinicians to meet the high demand for its palliative care services [88]. The plan addressed multiple challenges posed by the surge in COVID-19 cases: high numbers of severely ill patients, limitations on personal protective equipment, increased communication needs due to visitor restrictions and uncertainty about the novel disease, and restrictions on doctors' in-person field visits [88].

With aging populations and advances in science and technology, an increasing number of people diagnosed with life-limiting diseases will face longer periods of palliative care, which may require health care support for a period from six months to a year [89]. Some patients with terminal cancer wish to go to a memorable place or return home. However, owing to various symptom burdens and physical dysfunction, these wishes are difficult for them to realize [90]. VR can simulate physical locations and can hence be employed in facilitating a good death by allowing patients to have experiences on their “bucket list”, such as visiting the North Pole to see the aurora [90]. Likewise, as most patients do not wish to die in a hospital and would prefer the comfort of their home and company of their loved ones, patients can choose their ideal location of care during their last days using VR [90]. Research has shown that such virtual tours can improve spiritual wellbeing, physical and psychological symptoms, and blood pressure measurements in patients with advanced cancer [91].

There is growing evidence that VR is a positive psychological intervention for patients with advanced cancer receiving palliative care [92], with excellent analgesic effects [93]. Studies have demonstrated that this approach positively impacts the quality of life, mood, and health of adults receiving palliative care [94, 95], with significant improvements in pain, depression, anxiety, wellbeing, and shortness of breath [96]. The combination of VR and palliative care is not just for adults; it is also a way to help pediatric patients with serious medical conditions virtually leave their rooms while undergoing palliative care and improve their feelings of isolation [97]. This not only improves their nausea and headaches but also improves their mood [97].

In conclusion, virtual palliative care consultation is a promising resource that can help safeguard our health system's ability to address unmet palliative care needs for critically ill patients, especially during a pandemic [85].

### 5.4. Tai Chi

TC is a popular Chinese mind-body exercise [7]. Several studies have demonstrated the positive effect of TC in individuals, such as reducing the risk of cardiovascular disease [98] or preventing falls among elderly people at high risk of falls [99]. The ongoing COVID-19 pandemic has confined seniors most at risk of infection to their homes, reducing their opportunities for physical activity and worsening their physical performance [100]. Motivated by these public health challenges, some studies have explored the possibility of combining VR with TC, hoping to help elderly individuals reduce falls and improve balance and mobility through the program [100]. In a previous study, the authors attempted to apply the VR technique with TC to induce and enhance concentration, learning ability, fun, and feedback for older adults with cognitive impairment [7]. The results showed that VR-based TC exercise had protective effects on cognitive and physical function and that a higher degree of program participation was associated with greater improvements in cognitive performance [7]. The rapid conversion of TC programs from face-to-face to virtual classes has been feasible during the COVID-19 pandemic [101].

### 5.5. Qigong

Qigong is a mind-body therapy that has been widely used for health promotion and disease prevention in ancient China and India for thousands of years [102]. VR technology can be used to show the specific details of qigong movements in a complete view so that the recipient can observe more clearly and learn [8]. In VR, the actions of the recipient in the VR scene can be recorded and played back. This function allows the communicator to accurately assess whether the recipient's actions are standard through the recipient's specific actions and the data of the computer system and improve the teaching quality of online courses [8]. In addition, VR can affect the sensory system through sight, touch, hearing, etc. It can help individuals concentrate on life and achieve an optimal state in which the body, qi, and spirit are unified [8].

### 5.6. Acupoint Sticking Therapy

Acupoint sticking therapy is a treatment that works through the external application of a herbal paste, which is made from different materials according to the treatment purposes [103]. A study found that the use of acupoint sticking therapy combined with VR in children after circumcision effectively relieved their anxiety, diverted their attention, improved their pain perception threshold, and reduced their feelings of pain while also being noninvasive [6]. Acupoint sticking uses external treatment based on traditional Chinese medicine to relieve the physical discomfort of children, and VR uses three-dimensional dynamic vision and an interactive virtual world to divert the attention of children and provide a pleasant spiritual experience [6]. The two methods are easy to operate and are inexpensive. Due to the pleasant spiritual experience, the children in the intervention group were more cooperative in the follow-up nursing procedures, which not only improved the parents' and children's satisfaction with nursing care but also facilitated routine postoperative nursing procedures [6].

### 5.7. Aromatherapy

Aromatherapy, also known as essential oil therapy, is a complementary treatment that uses ingredients from different parts of plants, such as leaves, flowers, and seeds, to yield aromatic essential oils using different extraction techniques. Aromatherapy is widely used clinically in the treatment of postoperative nausea and vomiting [104] and dementia [105]. Research shows that the combination of 3D VR and hands-on aromatherapy allows for a powerful learning experience and facilitates the construction of a 3D space for aromatherapy products [4]. After 9 weeks of intervention, older subjects showed significant postintervention improvements in comparison with the control group in terms of the scores for happiness, perceived stress, sleep quality, meditation experience, and life satisfaction [4]. Additionally, this approach was found to increase the social participation and interpersonal communication of elderly people and reduce the waste of materials from hands-on activities [4].

### 5.8. Yoga

Yoga is a mind-body intervention that incorporates physical postures, breathing, and meditation to increase flexibility and strength, relaxation, and body awareness [106, 107]. Research found that VR-based yogic pranayama and meditation among health care workers was feasible during the COVID-19 pandemic and helped them feel more at peace, hopeful, and relaxed after the practice [9]. In a pilot study, participants preferred to engage in virtually delivered yoga interventions over face-to-face yoga, likely because it eliminated travel barriers and the risk of COVID-19 infection [108].

### 5.9. Comprehensive Application

Mind-body interventions such as relaxation, hypnosis, meditation, and music interventions for cancer patients who experience pain, fatigue, and sleep disturbances helped patients manage all symptoms in a group with a single treatment strategy [109]. In one study, subjects were offered mind-body group therapy sessions in fitness, meditation, yoga, dance, TC, and music using Zoom video conferencing during a COVID-19 outbreak [110]. The high utilization of and satisfaction with these virtual mind-body services demonstrate the significant potential of remote delivery to facilitate patient access to services [110]. A similar pilot study conducted in palliative care, where patients created a personalized soundtrack with a music therapist and then paired the soundtrack with a 360° VR environment, was well-rated by most participants, who described pleasant emotional and physical responses [111].

In summary, during a pandemic, a positive attitude and regular exercise are considered a strategy to strengthen the immune system to fight COVID-19 infection [112]. People can use VR systems combined with TC, qigong, yoga, etc., to facilitate exercise. Similarly, people can use VR with meditation, hypnosis, music therapy, and aromatherapy to help themselves relieve anxiety and panic caused by long-term isolation. At the same time, the combination of VR and meditation, hypnosis, palliative therapy, and acupuncture has become a necessary addition in CAM.

## 6. Teaching

### 6.1. Virtual Ward Rounds and Hospital Rotations

The COVID-19 pandemic has resulted in unprecedented public health measures. A survey of UK medical students showed that the impact on medical student education has been significant, particularly affecting the transition from a student to a doctor [113]. Limited exposure to medical school specialties has been shown to increase the likelihood of future medical mismanagement and misdiagnosis [114]. Therefore, given the uncertainty about the duration of the pandemic and the possibility of additional quarantine periods in the future, educational innovations are needed to ensure that medical students continue to be immersed in clinical settings.

Given the uncertainties about COVID-19, it is expected that students will continue to be excluded from evaluating COVID-19 patients in the near future. However, the COVID-19 pandemic has provided important teaching moments. How can educators provide medical students with first-hand knowledge of caring for COVID-19 patients while mitigating the risk of infection and addressing concerns about limited supplies of PPE [13]? Hoffman et al. explored the use of virtual ward rounds for medical students to observe and interact with COVID-19 patients to successfully educate students about the diagnosis and treatment of COVID-19 while eliminating the risk of infection [13].

During the COVID-19 pandemic, many universities and hospitals around the world, including the University of California, Los Angeles [22], Baylor College of Medicine [23], the University of Chicago [18], the Columbia University Irving Medical Center [15], and the University of Pennsylvania [11], have conducted similar experiments. After virtual hospital practicums, students appreciated the interactive nature of the course, felt that the instruction and rotation provided sufficient experience and confidence to understand internal medicine in a hospital setting, and expressed that they cherished this exposure to future career opportunities [11, 15, 18, 22, 23].

While helping students gain clinical knowledge, the virtual practicum approach reduces the burden on the health care system [115]. For example, Imperial College London uses this model to provide an effective triage system [16]; Harvard Medical School has developed the use of a virtual medical student response team of 500 students to educate or help a community or health care team [19]. Because of their positive role in helping during a pandemic, students report feeling empowered and enthusiastic, and they felt a sense of purpose during uncertain times. Additionally, the project promotes teamwork skills and indirectly increases students' knowledge and awareness of COVID-19.

Virtual practicums are a novel and successful model to help students familiarize themselves with the clinical environment, understand the mechanics of medical procedures, and help reduce health care burdens as COVID-19 continues to evolve. New interactive forms of virtual teaching are being developed to enable students to interact with patients from their homes. Open-access teaching with medical experts has enabled students to remain abreast of the latest medical advancements and to reclaim knowledge lost due to the suspension of university classes and clinical attachments [116]. At the same time, this virtual traineeship mitigates high rotation costs and removes financial barriers for all students [22]. Therefore, as COVID-19 continues to evolve and health systems respond, virtual internships and rotations are reasonable alternatives to in-person clinical rotations.

However, to some extent, inequalities in virtual teaching services worldwide are also noted to cause differences in medical education [116]. In developed countries such as the United Kingdom and the United States, the virtual teaching of medical students is a highly respected teaching method [16, 19]. In stark contrast, due to insufficient funds and infrastructure for virtual learning, some developing countries are yet to develop these teaching methods.

### 6.2. Teaching in Acupuncture

Acupuncture treatment, a traditional Chinese medical technology, is an extensive and rich practice, and teaching of acupuncture includes the teaching of human medicine, traditional medicine, acupuncture treatment methods, and clinical pain treatment [117]. In Chinese medicine, acupuncture points are of great significance to the human body and are an important part of learning acupuncture treatment techniques. The acupuncture points of the human body are identified through long-term observation and practice. They are special points on the surface of human organs, which serve as stimulation sites during acupuncture treatment. The acupoints of the human body are not only on the body's surface; their locations are deeply connected with the internal tissues and organs and are closely connected throughout the body [117].

At present, in most lessons on the position of acupoints, teachers use two-dimensional models such as pictures and multimedia software or use auxiliary teaching aids such as meridian and acupoint human models. Practical teaching regarding the position of acupoints generally includes finding the anatomical location of the acupoints on the body and drawing the direction of the meridians, etc., mainly relying on the students to practice on each other as operation subjects. However, the details cannot be viewed, and accuracy is lacking, which complicates the entire learning process [117]. The application of modern human anatomy knowledge in acupuncture makes the positioning of acupoints more standardized, but all Chinese medical schools have limited cadaveric resources, which has an impact on the development and quality of teaching. In the practice of acupuncture and moxibustion, in addition to practicing on themselves or other students, students often practice with paper balls, cotton balls and other substitutes [17]. This approach has no advantage in the three-dimensional sense of the meridians in the teaching display, and the students' experience is not strong in practice.

In response to these difficulties, some researchers have combined VR technology with anatomy [12, 24, 48] and applied it to the field of acupuncture teaching, aiming to create a virtual three-dimensional space to show the anatomical structure of acupuncture points to beginners in acupuncture and moxibustion, to realistically imitate the acupuncture process and to provide acupuncture points for these practices. This provides a safe and solid foundation to improve the efficacy of clinical acupuncture.

In a teaching experiment at Guangzhou University of Traditional Chinese Medicine, teachers used a virtual acupuncture teaching system to display the outline of the fourteen meridians and the local anatomy of the key points of each meridian (bones, blood vessels, nerves, muscles, and epidermal texture) [17]. When teaching acupuncture and moxibustion procedure courses, the virtual acupuncture teaching system can be used to construct intelligent three-dimensional animations, which vividly display the needle insertion level of each acupoint and the danger of an incorrect acupuncture procedure [17]. When students practice the operation, the system displays the hierarchical anatomical structure according to the needle insertion level in virtual acupuncture. If the acupuncture is wrong, the system will give a prompt response, and the score of the operation will be displayed after the acupuncture procedure is completed [17]. This fun and interactive learning method not only improves test scores but also improves students' enthusiasm for learning [17].

In VR, adding tactile feedback to simulate the sense of touch in the real world to visual feedback can greatly enhance the operator's sense of reality [14]. Through a force-feedback device, Jiang Jun et al. collected acupuncture experts' Fengchi acupuncture techniques, integrated them into a digital virtual human body, and used VR technology to build a virtual Fengchi acupuncture force-feedback simulation system so that the operator could achieve one-to-one acupuncture. The advanced simulation learning effect can simulate the visual, tactile, and force sensation of needle insertion to achieve the purpose of rapidly improving the learner's acupuncture skills, which helps in transferring traditional Chinese medicine skills from a virtual anatomical person to a real physical person [14].

### 6.3. Teaching in Palliative Care

Dying patients are a reality in medicine [20]. As the population ages, more knowledge, skills, and experience in palliative care are needed to manage end-of-life patients. Medical students, however, feel unprepared to effectively navigate the complex end-of-life management issues of dying patients and want increased experiential learning in palliative care [20]. In teaching students in palliative care, VR technology proves to be an effective teaching tool that may help address the need to add formal palliative care experience to medical school training programs [20, 21].

Palliative care, on the other hand, is often delivered by an interdisciplinary team through different hospital stages to address the needs of patients and families; the team often includes advanced practice nurses, physicians, registered nurses, social workers, and spiritual or religious counselors. The team may also include members from other health care professions, including nutrition, physical therapy, and occupational therapy [118]. The use of VR technology could be an important way for palliative care courses to effectively and conveniently help students from different majors meet on a certain day, time and place, bringing interprofessional learners together [26].

## 7. Scientific Research

### 7.1. Virtual Diagnosis

Using an online virtual diagnostic model to determine the association between the diagnostic model and the designated acupoints is a new research method for acupoints. In one study [26], acupuncture practitioners were asked to participate in a virtual diagnosis process, a method employed in previous studies to evaluate the performance of doctors and medical students [119, 120]. According to the model data, the model could evaluate the commonality and specific treatment prescription of various acupoint selections and explore the core acupoints for specific diseases [26]. Kyung Hee University also conducted a similar study [25]. Based on the virtual diagnoses of currently practicing doctors, the results suggested a relationship between symptom indications and acupoint prescriptions in Korean medicine and revealed clear patterns of acupoints commonly prescribed across various diseases, as well as acupoints used in specific cases [26].

This study had several limitations that should be considered [26]. First, due to the nature of the experiment, the validity of virtual diagnoses could not be assessed, and it is necessary to review other types of data to support this [121]. Second, prospective studies should include a larger sample including physicians from around the globe to cover the wide range of different skills among physicians [121].

## 8. Advantages of Using VR for CAM

There are numerous benefits of using VR over traditional methods. In determining whether the combination of VR and CAM is ready for widespread use, we need to consider what capabilities VR offers that make it particularly suitable for clinical practice, teaching, and scientific use in the field of CAM. On a very broad level, VR can facilitate the development of individual therapies in the field of CAM. These aids can be summed up simply as follows.

First, this review found convincing evidence that VR has widespread clinical use. VR eliminates a potential barrier for patients who may experience difficulty imagining or visualizing. VR can enhance therapy by enhancing sensory immersion (e.g., VR combined with meditation therapy can help patients maximize immersion, and VR provides compelling visual and auditory stimuli in people with low hypnotic susceptibility). Simultaneously, virtual locations can be simulated to transport the patient to where he or she wants to go. For example, VR can help patients who are receiving palliative care to fulfill their wishes to travel or return home. It can also help people practicing yoga, qigong, TC, etc., at home to pretend they are in a classroom. These exercises are embedded in sports or games and are more engaging than staying home all the time. Moreover, interactivity should be used to help palliative care patients in hospitals make real-world connections with loved ones.

Second, in teaching, VR can help medical students with virtual medical practice during the COVID-19 pandemic. In some special disciplines, such as acupuncture and palliative care, VR plays an irreplaceable role. More importantly, VR can provide behavioral performance capture and retrospective and intuitive post hoc evaluation. Safe testing and training environments minimize the risks due to errors.

Third, VR introduces a new method and opens new avenues for overcoming boundaries in scientific CAM research.

Fifth, from a research perspective, the use of VR could facilitate data collection during the COVID-19 pandemic to monitor progress, providing policymakers with valuable information such as factors affecting the disease course, infectivity, and disease severity.

Sixth, VR can reduce infection rates and health care burdens. Especially for patients with reduced mobility, a VR headset can be used safely in the patient's home, which can reduce the need for hospital visits [122]. In teaching, the use of VR may allow simple tasks in clinical practice to be repeated multiple times in an immersive environment without constant supervision by medical staff, which could significantly reduce the cost of training facilities and trained medical staff [122].

In conclusion, the application of VR in CAM has great scientific, practical, and socioeconomic implications that can help people stay healthy and reduce the burden on the health care system.

## 9. Limitations of VR-Based CAM and Recommendations for How to Improve

Unfortunately, many challenges need to be overcome before this vision of clinical VR can be achieved. Setting up VR systems in clinical settings remains technically challenging and costly, requiring ongoing technical assistance, skill development, and infrastructure investment, which is especially challenging in resource-constrained settings [123]. While the initial cost of using VR continues to be a potential disadvantage, prices have decreased over time. As VR-enabling technologies and methods continue to evolve, the widespread adoption of VR in the CAM space will likely involve more advanced, less expensive systems and will be generally welcomed.

While conducting scientific research in CAM with VR, problems have been noted, including small sample sizes, a lack of methodological rigor, and lack of comparison groups. When designing a VR study, the use of a control condition and large enough sample sizes for sufficient power to detect an effect while considering possible treatment drop-out rates and projected attrition over all follow-up assessments are recommended [38]. A need exists for more well-powered and controlled studies comparing VR-based treatments to other treatments, including real-world medical records, randomized clinical trial data, and traditional medical texts.

## 10. Summary and Outlook

We previously assessed the acceptability of VR for hospitalized patients and found that most patients found the use of VR to be a positive and pleasurable experience, relieving anxiety and providing a form of escape from the confines of distressing illness experiences. Most patients reported that they would be willing to use VR again if given the opportunity.

The COVID-19 pandemic has accelerated the implementation of video- and audio-capable telemedicine infrastructures around the world. The advancement and widespread acceptance of these virtual communication technologies is a clear trend in the current pandemic. Clinicians, medical students, and researchers have had to adapt quickly to using a combination of VR and clinical applications, and in most cases, it works well.

As we have discussed, VR enables the better development of CAM in dynamic, complex, and realistic situations. VR methods continue to accrue validating results. This trend should continue as these methods become widely adopted and are extended to the study of different areas and a wider range of therapies.

However, despite rapid development, this relatively new field calls for replication and standardization as part of a theoretical framework to facilitate reflective, purposeful progress that is not driven solely by technology [33]. Training programs in CAM should also encourage students to consider how VR and other technological advances can better help us serve our patients and the public.

Going forward, we should continue to build on the positive contribution of VR to the field of CAM.
